# Systematic Nursing Interventions Combined with Continuity of Care in Patients with a Spinal Fracture Complicated with a Spinal Cord Injury and Its Effect on Recovery and Satisfaction

This article has been retracted.

**DOI:** 10.1155/2022/3771144

**Published:** 2022-08-05

**Authors:** Yingjie Xia, Jing Wang, Ping Wang

**Affiliations:** ^1^Department of Orthopedics, Affiliated Hospital of Jiangnan University, Wuxi, Jiangsu Province, China; ^2^Department of Orthopedics, Nantong First People's Hospital, Nantong 226001, Jiangsu Province, China

## Abstract

**Objective:**

The aim of this study is to examine the application value of systematic nursing interventions combined with continuity of care in cases with a spinal fracture complicated with a spinal cord injury and its effect on recovery and satisfaction.

**Methods:**

We identified ninety cases with a spinal fracture complicated with a spinal cord injury who were admitted to local hospital from May 2019 to May 2021 as research subjects and assigned them into an experimental group (systematic nursing combined with continuity of care, *n* = 45) and a control group (conventional nursing, *n* = 45) according to their admission order. The level of life of all groups between intervention was evaluated with reference to the Generic Quality of Life Inventory-74 (GQOLI-74) Rating Scale. The Hospital Anxiety and Depression (HAD) scale was used to assess the emotional status of patients before and after intervention. The complication rates, nursing outcomes, nursing satisfaction, and rehabilitation outcomes of all cases were calculated.

**Results:**

The GQOLI-74 score of the experimental group was higher than that of another group (*P* < 0.05). Lower HAD scores of experimental group were observed than that of another group (*P* < 0.05). The experimental group obtained remarkably higher nursing effective rates and higher nursing satisfaction than another group (*P* < 0.05). Rehabilitation outcome of the experimental group outperformed that another group (*P* < 0.05).

**Conclusion:**

The use of systematic nursing intervention combined with continuity of care for cases with spinal fracture complicated with a spinal cord injury can enhance the nursing effect, effectively relieve cases' psychological pressure, improve patients' level of life and nursing satisfaction, and contribute to the maintenance of a good nurse-patient relationship, which merits clinical promotion.

## 1. Introduction

Spinal fracture complicated and spinal cord injury is a common traumatic disease in clinical practice, which can lead to dysfunction of the body, a variety of complications, negative emotions in the patients, severely compromising their level of life and mental health. If the spinal fracture is associated with spinal cord injury, the main complication is a reduction or even loss of sensory movement in the limbs; if it occurs in the cervical or thoracic spine, it is accompanied by urinary and faecal dysfunction; if it occurs in the lumbar spine, the main complication is a loss of sensory movement in both lower limbs. If the spinal cord injury occurs, the patient is bedridden for a relatively long period of time, which can easily lead to bed sores, pneumonic pneumonia, and urinary tract infections [1–3]. If the patient has underlying medical conditions, such as hypertension and hyperlipidaemia, this may also lead to venous thrombosis of the lower limbs, or even heart attack, cerebral infarction, or pulmonary embolism, which can seriously affect the patient's quality of life and even threaten the patient's life [4, 5]. Therefore, effective care measures are required for patients with spinal fractures with a spinal cord injury [6–8].

Systematic care is a new scientific, targeted, systematic, and patient-centred care model. Preoperative and intraoperative care for patients can effectively alleviate negative emotions such as fear, depression, and anxiety, reduce patients' psychological burden, maintain a positive surgical mindset, and ensure smooth surgery, while postoperative care for patients can help reduce the incidence of complications and promote recovery. However, nursing care for patients only during hospitalization fails to ensure a satisfactory nursing outcome. Therefore, continuity of care is introduced to patients after discharge, with targeted rehabilitation training for patients to improve their quality of life and relieve negative emotions, which can effectively shorten their rehabilitation time and further accelerate their recovery [9–11]. The continuum of the care model has been applied to chronic diseases in the elderly with good results; furthermore, some studies have found its application in the recovery process of other diseases as well [12]. Accordingly, 90 cases with a spinal fracture complicated with a spinal cord injury were included to examine the application value of systematic nursing interventions combined with continuity of care in cases with spinal fracture complicated with a spinal cord injury, its influence on recovery and satisfaction. The report is as follows.

## 2. Materials and Methods

### 2.1. General Information

Ninety cases of spinal fracture combined with spinal cord injury in our hospital between May 2019 and May 2021 were identified as subjects, assigned into an experimental group (*n* = 45) and a control group (*n* = 45) according to their admission order.

### 2.2. Inclusion Criteria

The inclusion criteria were as follows: (1) those with abundent clinical data; (2) cases with significant history; (3) cases with single-segment spinal fractures; (4) those with the ability to communicate and clear consciousness; and (5) the study was approved by Medical Ethics Committee, both cases and patients' families signed consent forms with knowledge of the study.

### 2.3. Exclusion Criteria

The exclusion criteria were as follows: (1) those with acute infection or chronic infection; (2) those with symptoms of paralysis prior to fracture; (3) those with abnormal blood count and abnormal coagulation mechanism; (4) those who cannot tolerate surgery; and (5) those with psychiatric disorders.

### 2.4. Methods

The control group included reasonable diet guidance (According to *People's Republic of China Health Industry Standard* No.: WS/T558-2017) and rehabilitation training plan [13].

Patients in the experimental group were given systematic nursing interventions combined with continuity of care.

1. Upon admission, the nursing staff will provide education on the case and an introduction to the hospital environment to help them fully understand the disease-related knowledge and ease their unfamiliarity with the hospital environment.
2. The nursing staff informed the patient of the procedure and the significance of the surgery beforehand and provided psychological interventions to alleviate the patient's nervousness and fear. The nursing staff formulated care plans in conjunction with the patient's surgical and anaesthetic protocols to ensure that the operating theatre was at the right temperature, adequately lit, adequately prepared for blood transfusion, and adequate surgical instruments. Emergency plans were formulated in advance to avoid unexpected events during surgery.
3. The patients were instructed to perform abdominal respiration which could reduce the risk of oxygen aspiration in case of intraoperative respiratory distress due to pain and spinal nerve injury. The nursing staff closely monitored the patient's vital signs and also promptly assessed the condition of the external fixator. Abnormalities in the patient's vital signs require immediate cooperation with the physician to perform appropriate treatment measures.
4. Postoperative nursing staff closely monitor the patient's oxygen saturation, blood pressure, and electrocardiogram (ECG) signals. We secure the patient's drainage tube and catheter to prevent blockage and bending of the tube. We record in detail the volume, colour, and nature of the patient's drainage fluid [10, 11, 14].
5. The patients were provided with reasonable dietary instruction, including intake of easily digestible foods, a daylong stream of mini-meals, and prohibition of spicy foods.
6. A one-month follow-up was conducted after discharge, and the nursing staff recorded in detail the recovery of the patients, actively communicated with the patients and their families, and endeavored to help solve the patients' difficulties. The nursing staff advised the family members to actively encourage the patients to reduce their psychological burden and relieve their negative emotions, which is conducive to enhancing the patients' compliance with treatment and enabling them to better accept nursing treatment.
7. The nursing staff formulated rehabilitation schemes for the patients and provided guidance on their rehabilitation training. It was necessary for the patient to be turned over every two hours and to be massaged by 2–3 times a day which was performed by the family, to effectively avoid stiffness of the patient's joints. After the condition has been improved, the patients were instructed to carry out training such as sitting, standing, and walking according to their actual condition, adhering to the principle of gradual progress, to enhance their self-care ability.
8. Potential complications need to be prevented, as they may hinder recovery or even threaten the patient's life. During hospitalisation, patients are instructed by nursing staff to perform appropriate coughing and breathing exercises, and their families are instructed to assist in turning the case to avoid pressure sores and to pat the patient's back at home for sputum evacuation [15–18].
9. Nursing staff carried out family education to the patients and their families as the family environment might affect the patients' recovery. Therefore, during the recovery, the patients' families should maintain a positive attitude and actively carry out rehabilitation training with the patients, which can effectively accelerate the patients' recovery.

### 2.5. Observational Indicators

Incidence of complications was compared between all groups of patients. Complication rate = number of people with complications/total number of people in the group × 100%.

The level of life of the two groups of cases before and after nursing was evaluated with reference to Generic Quality of Life Inventory-74 (GQOLI-74) rating scale [19], which scores four scoring factors from psychological function, physical function, social function, and scores range from 76 to 380 points. The higher the score, the better the quality of life.

Hospital Anxiety and Depression [20] (HAD) scale was used to assess emotional state of patients before and after intervention, with a total score of 42 on this scale (scores range from 0 to 21 for anxiety and 0 to 21 for depression). Higher level represent more severe anxiety and depression in patients. 8–10 is mild, 11–14 is moderate, and 15–21 is severe [21].

Comparison of nursing outcomes between all patients [1]. Significantly effective: Significant improvement in clinical symptoms and return of consciousness within 12–24 hours of care, no complications. Effective: clinical symptoms resolved within 12–24 hours of care, recovery of consciousness, minor complications. Ineffective: no improvement in clinical symptoms, no recovery of consciousness and serious complications within 12–24 hours of care. (Effective number + effective number)/total number *∗* 100% = total effective rate.

### 2.6. Statistical Analyses

SPSS20.0 was used to statistically process the data and GraphPad Prism 7 (GraphPad software, San Diego, USA) was used to draw the graph. *χ*2 test was performed on the count data, which was expressed as (*n* (%)), and the measurement data were expressed as (*n* (%)) (*x* ± *s*) and analyzed by *t*-test. *P* < 0.05 indicates that the difference is significant.

## 3. Results

### 3.1. Comparison of General Information

Two groups showed no difference in general information such as BMI, smoking, drinking, and place of residence (*P* > 0.05). See Table 1.

### 3.2. Comparison of the Incidence of Complications

In the experimental group, 2 individuals had healing deformities (4.44%), 1 individual had a decubitus ulcer (2.22%), 1 individual had constipation (2.22%), and none had an infection (0.00%), for an overall complication rate of 8.89%; in the control group, 6 individuals had healing deformities (13.33%), 5 individuals had decubitus ulcers (11.11%), 4 individuals had constipation (8.89%), and 3 had an infection (6.67%), for an overall complication rate of 40.00% ( 8.89%), 3 infections (6.67%), and an overall complication rate of 40.00%. the experimental group had a lower complication rate compared with that of another group (*P* < 0.05). See Table 2.

### 3.3. Comparison of the GQOLI-74 Score

The GQOLI-74 scores before and after the intervention were (46.44 ± 7.88) and (82.33 ± 4.98), respectively, for the experimental group; the GQOLI-74 scores before and after the intervention were (46.72 ± 7.43) and (61.25 ± 4.22), respectively, for the control group. Higher GQOLI-74 scores were observed in the experimental group as compared to those of another group (*P* < 0.05). See Figure 1.

### 3.4. Comparison of the HAD Score

The HAD scores of (35.81 ± 3.25) and (5.36 ± 1.21) before and after the intervention for patients in the experimental group; HAD scores of (35.88 ± 3.22) and (13.29 ± 2.53) before and after the intervention for patients in the control group, respectively. The experimental group obtained markedly lower HAD scores than another group (*P* < 0.05). See Figure 2.

### 3.5. Comparison of Nursing Outcomes

In the experimental group, the apparent efficiency was 68.89% (31/45), the effective rate was 28.89% (13/45), the inefficiency was 2.22% (1/45), and the total effective rate was 97.78% (44/45); in the control group, the apparent efficiency was 51.11% (21/45), the effective rate was 35.56% (16/45), the inefficiency was 17.78% (8/45), and the total effective rate was 82.22% (37/45). The total effective rate was 82.22% (37/45). A higher effective rate was recorded in experimental group in contrast to that of another group (*P* < 0.05). See Figure 3.

### 3.6. Comparison of Nursing Satisfaction

In the experimental group, the satisfaction rate was 71.11% (32/45), the moderate satisfaction rate was 22.22% (10/45), the dissatisfaction rate was 6.67% (3/45), and overall satisfaction rate was 93.33% (42/45); in the control group, the satisfaction rate was 44.44% (20/45), the moderate satisfaction rate was 28.89% (13/45), the dissatisfaction rate was 26.67% (12/45), and overall satisfaction rate was 73.33% (33/45). (12/45), with an overall satisfaction rate of 73.33% (33/45). The experimental group obtained higher nursing satisfaction rate in comparison with other group (*P* < 0.05). See Figure 4.

### 3.7. Comparison of Rehabilitation

A superior rehabilitation outcome was observed in the experimental group compared to that of another group (*P* < 0.05). See Table 3.

## 4. Discussion

Spinal fractures are a common type of fracture in clinical practice and are often complicated by a spinal cord injury. The high incidence and severity of this condition can also disrupt the environment within the patient's vertebral body and spinal canal, making surgical treatment very difficult and high-risk due to the complex anatomy of the tissues surrounding the spine. Surgery is the primary treatment for spinal fractures combined with spinal cord injury. It helps to restore neurological function by decompressing the spinal canal, relieving spinal cord compression, correcting spinal deformities and effectively improving spinal stability. However, surgical treatment can only serve to eliminate spinal cord compression symptoms, and patients' limb activity will be restricted after surgical treatment which requires long-term bed rest. Moreover, the risk of different degrees of physical disability may result in negative emotions and thus psychological problems in patients [22–24], for which conventional nursing fails to yield a satisfactory outcome. For example, cerebrospinal fluid leakage is a frequent complication after spinal fracture surgery. Due to compression and adhesion of the fracture fragment to the dura mater, a tear in the dural sac may result when decompression is performed to separate the fracture fragment, and a tear in the dural sac that is incompletely sutured, or a large tear that is not easily sutured and not repaired in time can result in cerebrospinal fluid leakage [25–27]. One of the most serious consequences of a cerebrospinal fluid leak is a retrograde intracranial infection [27]. In the case of spinal fractures, especially in the cervical and thoracic segments, the process of decompression of the spinal cord may cause secondary damage to the spinal cord or nerves, which may result in secondary paralysis, aggravation of existing paralysis, or even an increase in neurological impairment [28].

Conventional care has failed to produce satisfactory outcomes and reasonable and effective nursing interventions are needed to improve the patient's recovery and standard of living. In systemic care, nursing staff develop systematic care measures for patients based on a comprehensive understanding of their actual condition. It has been noted that applying systemic care to patients with spinal fractures combined with spinal cord injury can reduce the incidence of complications in cases and further reduce their clinical symptoms [29–32]. Continuity of care is the extension of care from in-hospital nursing to home nursing. Nursing staff develop care schemes for patients and guide patients' family members with regard to home care to ensure a better home care quality and rehabilitation training outcome. A study by (2019) showed that continuity of care for cases can effectively improve the adverse mood of depression and anxiety, and psychological care for patients relieves their negative emotions and their psychological burden [33]. This study demonstrated that quality of life of experimental group was better than another group (*P* < 0.05), which is consistent with findings of who stated in their article that “the GQOLI-74 score of the observation group was (84.56 ± 2.13), which was significantly higher than that of (63.54 ± 2.67) of the control group,” indicating that in comparison with conventional nursing, systematic nursing interventions combined with continuity of care can efficiently boost the patients' quality of life, enhance their clinical symptoms and prominently relieve their negative emotions [34].

Spinal cord injury is the most serious complication of spinal injury, enough to cause severe dysfunction of the limbs below the injured segment. In Chinese medicine, it is mostly seen in the category of impotence and should be treated with evidence-based medicine [35, 36]. For those with weakness of both lower limbs, muscle atrophy, fatigue, lack of breath and speech, reduced diet, diarrhoea and loose stools, etc., they can follow medical advice to choose drugs that tonify the middle and vital energy, strengthen the spleen, and promote clearing [37, 38]. For those who manifest impotence and weakness of both lower limbs, complete paralysis, muscle atrophy with dizziness and tinnitus, dry throat and tongue, etc., consider liver and kidney deficiency, and choose drugs to nourish the liver and kidney, nourish Yin, and clear heat [37, 38]. For patients with high paraplegia can be treated by physical methods such as massage physiotherapy tui-na and acupuncture, which can help improve the symptoms and stabilize the condition, and can play a certain therapeutic role [39].

In conclusion, the use of systematic nursing intervention combined with continuity of care for cases spinal fracture and spinal cord injury can enhance the nursing effect, reduce incidence of complications, effectively relieve cases' psychological pressure, improve patients' level of life and nursing satisfaction, and contribute to maintenance of a good nurse-patient relationship, which merits clinical promotion. However, the experiment only explored this area of spinal fracture combined with spinal cord injury and we still need to think about whether the combination of systematic care and continuous care is equally effective for different conditions. On this basis, we can continue to innovate in our care protocols by adding specialist care approaches for different departments, combined with effective Chinese medicine, which is something we need to continue to explore in the future.

## Figures and Tables

**Figure 1:** Comparison of the GQOLI-74 score between the two groups of patients (*x* ± *s*). The abscissa represents before and after intervention, and the ordinate represents GQOLI-74 score points. The GQOLI-74 scores of patients in the experimental group before and after intervention were (46.44 ± 7.88) points and (82.33 ± 4.98) points, respectively; The GQOLI-74 scores of the control group before and after intervention were (46.72 ± 7.43) points and (61.25 ± 4.22) points, respectively; ^*∗*^indicates that there is a significant difference in the GQOLI-74 scores of the experimental group before and after intervention (*t* = 25.828, *P* < 0.05); ^*∗∗*^indicates that there is a significant difference in the GQOLI-74 scores of the control group before and after intervention (*t* = 11.407, *P* < 0.05); ^*∗∗∗*^indicates that there is a significant difference in GQOLI-74 scores between the two groups of patients after intervention (*t* = 21.663, *P* < 0.05).

**Figure 2:** Comparison of the HAD score between the two groups of patients (*x* ± *s*). The abscissa represents the pre-intervention and post-intervention, the ordinate represents the HAD score points. The HAD scores of the patients in the experimental group before and after intervention were (35.81 ± 3.25) points and (5.36 ± 1.21) points, respectively; The HAD scores of the control group before and after intervention were (35.88 ± 3.22) points and (13.29 ± 2.53) points, respectively; ^*∗*^indicates that there is a significant difference in the HAD scores of the experimental group before and after intervention (*t* = 58.901, *P* < 0.05); ^*∗∗*^indicates that there is a significant difference in the HAD scores of patients in the control group before and after intervention (*t* = 37.005, *P* < 0.05); ^*∗∗∗*^indicates that there is a significant difference in the HAD scores of the two groups of patients after intervention (*t* = 18.968, *P* < 0.05).

**Figure 3:** Comparison of nursing outcomes between the two groups of patients (*n* (%)). (a) The nursing effect of the experimental group. (b) The nursing effect of the control group. In the experimental group, the markedly effective rate was 68.89% (31/45), the effective rate was 28.89% (13/45), the ineffective rate was 2.22% (1/45), and the total effective rate was 97.78% (44/45). In the control group, the markedly effective rate was 51.11% (21/45), the effective rate was 35.56% (16/45), the ineffective rate was 17.78% (8/45), and the total effective rate was 82.22% (37/45). There is a significant difference between the two groups of patients after nursing (*X*2 = 6.049, *P* < 0.05).

**Figure 4:** Comparison of nursing satisfaction between the two groups of patients (*n* (%)). (a) The nursing satisfaction of the experimental group. (b) The nursing satisfaction of the control group. In the experimental group, the satisfied rate was 71.11% (32/45), the moderately satisfied rate was 22.22% (10/45), the dissatisfied rate was 6.67% (3/45), and the overall satisfaction rate was 93.33% (42/45). In the control group, the satisfied rate was 44.44% (20/45), the moderately satisfied rate was 28.89% (13/45), the dissatisfied rate was 26.67% (12/45), and the overall satisfaction rate was 73.33% (33/45). There is a significant difference between the two groups of patients after nursing (*X*2 = 6.480, *P* < 0.05).

**Table 1:** Comparison of general information between two groups of patients.

	Experimental group (*n* = 45)	Control group (*n* = 45)	*χ* ^2^ or *t*	*P*
*Age (years)*			0.086	>0.05
	36.75 ± 3.32	36.69 ± 3.29		

*Gender*			0.178	>0.05
Male	23 (51.11)	21 (46.67)		
Female	22 (48.89)	24 (53.33)		

*BMI (kg/m * ^*2*^)			1.119	>0.05
	26.27 ± 1.59	25.89 ± 1.63		

*SAS scores (points)*			0.451	>0.05
	48.12 ± 1.38	48.26 ± 1.56		

*SDS scores (points)*			0.112	>0.05
	51.24 ± 2.36	51.18 ± 2.73		

*Smoking*			0.045	>0.05
Yes	20 (44.44)	21 (46.67)		
No	25 (55.56)	24 (53.33)		

*Drinking*			0.178	>0.05
Yes	22 (48.89)	24 (53.33)		
No	23 (51.11)	21 (46.67)		

*Place of residence*			0.050	>0.05
Urban	31 (68.89)	30 (66.67)		
Rural	14 (31.11)	15 (33.33)		

**Table 2:** Comparison of the incidence of complications between the two groups of patients (*n* (%)).

Groups	*n*	Healing deformities	Pressure sore	Constipation	Infection	Total incidence
Experimental group	45	2 (4.44)	1 (2.22)	1 (2.22)	0 (0.00)	4 (8.89)
Control group	45	6 (13.33)	5 (11.11)	4 (8.89)	3 (6.67)	18 (40.00)
*χ* ^2^						11.971
*P*						<0.05

**Table 3:** Comparison of rehabilitation between the two groups of patients (*yx* ± *s*).

Groups	*n*	MBI	GSES	FIM
Experimental group	45	86.37 ± 2.14	32.76 ± 1.41	113.52 ± 9.83
Control group	45	73.56 ± 1.28	26.12 ± 1.35	99.62 ± 9.14
*T*		34.461	22.818	6.947
*P*		<0.05	<0.05	<0.05

## Data Availability

No data were used to support this study.
